The article "The Efficacy of Artificial Intelligence in the Detection and Management of Atrial Fibrillation" was retracted in 2026. Reasons: errors in the text; unreliable results or conclusions; concerns about the citations.

# The Efficacy of Artificial Intelligence in the Detection and Management of Atrial Fibrillation

**DOI:** 10.7759/cureus.77135

**Published:** 2025-01-08

**Authors:** Apurva Popat, Sweta Yadav, Jacob Obholz, Elliot A Hwang, Ateeq U Rehman, Param Sharma

**Affiliations:** 1 Internal Medicine, Marshfield Clinic Health System, Marshfield, USA; 2 Cardiology, Marshfield Clinic Health System, Marshfield, USA

**Keywords:** af prediction, ai ecg, ai in cardiology, artificial intelligence, atrial fibrillation, machine learning, wearable devices

## Abstract

The integration of artificial intelligence (AI) into medicine offers transformative potential, particularly in the detection and management of atrial fibrillation (AF). However, the intersection of AI and AF has not been comprehensively evaluated. This systematic review focuses specifically on the applications of AI in AF risk prediction, monitoring, and management. Following the Preferred Reporting Items for Systematic Reviews and Meta-Analyses (PRISMA) guidelines, a comprehensive search was conducted in PubMed and Google Scholar using terms such as artificial intelligence, deep learning, machine learning, artificial neural networks, and AF diagnosis. Methodological quality and risk of bias were assessed using the JBI critical appraisal checklist for qualitative research. Of the 109 studies screened, 39 met the inclusion criteria. Of these, 19 studies focused on AI’s role in AF risk prediction, while 20 studies addressed its application in monitoring and management. Machine learning models, including AI-ECG approaches such as the optimal time-varying machine learning model and the observational medical outcomes partnership common data model, demonstrated superior sensitivity and specificity compared to traditional models (Framingham, atherosclerosis risk in communities (ARIC), congestive heart failure, hypertension, age ≥75, diabetes, stroke, vascular disease (CHADS-VASc), and cohorts for heart and aging research in genomic epidemiology model for atrial fibrillation (CHARGE-AF). Wearable devices, such as patch monitors and smartwatches, emerged as reliable, cost-effective, and noninvasive alternatives to implantable cardiac monitors for continuous AF detection and patient-centered management. Despite these advances, the reliability and consistency of AI-based tools remain variable across studies due to data heterogeneity and methodological inconsistencies. Identified gaps include the need for standardized, labeled datasets, robust validation through prospective clinical trials, and improved data governance frameworks to ensure reliability and reproducibility. In conclusion, AI holds immense potential for AF prediction and management, but addressing these challenges is essential for its integration into clinical practice.

## Introduction and background

Atrial fibrillation (AF) is the most prevalent cardiac arrhythmia globally [1]. The global prevalence of AF is approximately 60 million cases, with significant associated risks including a 2.4-fold increase in stroke, 1.5-fold increase in dementia, 1.5-fold increase in myocardial infarction, and a 5-fold increase in heart failure [1,2]. Key risk factors include hypertension, obesity, coronary artery disease, and advanced age [1]. High-risk populations include the elderly, individuals with a history of cardiovascular disease, and those with comorbid conditions such as chronic kidney disease and diabetes [1].

Each year, graduating medical students are formally inducted into the medical profession, guided by well-defined ethical principles [3]. These principles, enshrined in national medical institution charters and regulatory frameworks, establish the foundation for clinical practice, and their violation constitutes medical malpractice [4]. The integration of AI into healthcare must align with these ethical principles: beneficence, nonmaleficence, autonomy, and justice to promote patient welfare, minimize harm, ensure informed consent, and provide equitable access to healthcare advancements [5]. While AI is increasingly applied in medical settings, its primary purpose must remain improving patient care and quality of life [6,7]. Achieving this requires high levels of accuracy in clinical applications, supported by advanced computational capabilities, such as high-performance computing, cloud computing, edge computing, and robust data management systems [6,7]. Recent technological advancements have made it possible to solve previously intractable problems efficiently, bringing the vision of seamless, effective, and equitable healthcare closer to reality.

Atrial fibrillation (AF) intervention practice has gracefully embraced the adoption of AI. The prediction of new cases is facilitated by predictive analytics [7]. Predictive analytics and modeling constitute various statistical methods such as Machine Learning (ML), data mining, and modeling that examine clinical patient data to predict the probability of future AF events [8]. The predictive models are trained with patient data from large electronic health records databases. The patient data might include comorbidities, family history, and demographics [6,9]. A risk score can then be developed for a specific patient and can be used to deliver personalized treatment and care [9]. As technology continues to improve amid the standardization and expansion of medical databases, the role of AI in patient management is expected to expand. For example, a study using a deep neural network (DNN) model to predict incident AF in post-stroke patients achieved a C index of 0.77, significantly outperforming traditional clinical scores such as congestive heart failure, hypertension, age ≥75 years, diabetes, and stroke (CHADS2), and congestive heart failure, hypertension, age ≥75years, diabetes, stroke, vascular disease (CHADS-VASc). Another study comparing a time-varying neural network model to traditional models found that the ML model achieved an area under the receiver operating characteristic curve (AUC) of 0.827, compared to 0.725 for the best existing model, cohorts for heart and aging research in genomic epidemiology model for atrial fibrillation (CHARGE-AF) [10,11].

Notably, AI can be integrated into inpatient and outpatient treatment of AF, with sufficient scope to deal with the specific risk profile of each patient [9]. Cardiological rehabilitation through an integrated approach provides the opportunity to establish individual, lifestyle-oriented risk management. AI-enabled wearables, such as smartwatches, ECG patches, and smart textiles, continuously monitor physiological parameters like heart rate and rhythm, providing real-time data for early detection and management of AF [6,12]. This leads to symptomatic improvement, decreased AF burden, enhanced performance, and a better quality of life [8,13]. Beyond standard treatments like anticoagulation, rate and rhythm control, and comorbidity management, modifying risk factors is probably the most critical element in improving patient outcomes [13]. Risk modification encompasses mitigating modifiable risk factors to prevent the development and progression of AF [14]. For example, AI can help manage blood pressure, weight, and other modifiable risk factors, leading to symptomatic improvement, decreased AF burden, enhanced performance, and a better quality of life [15].

Nevertheless, AI has potential risks. AI may be able to advance science and find solutions for complex problems, but there are accompanying unintended consequences [16]. These risks include data privacy and copyright infringement [6,17]. As such, AI training should incorporate ethics and bias attenuation. To mitigate risks like data privacy breaches, bias, and copyright infringement in AI-driven atrial fibrillation care, strategies such as diverse training datasets, adherence to findable, accessible, interoperable, and reusable (FAIR) data principles, compliance with regulations like health insurance portability and accountability act (HIPAA), general data protection regulation (GDPR), regular algorithm audits, and interdisciplinary collaboration are essential for ethical and effective implementation [18]. The purpose of this systematic review is to comprehensively analyze the literature, identify gaps and limitations, assess the efficacy of AI applications in AF, and provide evidence-based recommendations for guiding both clinical practice and future research, focusing on AI’s role in AF risk prediction, diagnostic tools, and management strategies.

## Review

Materials and methods

Literature Search and Reporting

This review was reported according to the recommendations of the Preferred Reporting Items for Systematic Reviews and Meta-Analyses (PRISMA) [19]. Literature searches were done using PubMed and Google Scholar. A supplementary bibliography search was also performed. The keywords used include artificial intelligence, deep learning, machine learning, artificial neural networks, and AF diagnosis (Table 1).

**Table 1:** Search strategies and databases used.

Database/tool	Search terms	Date of search	Filters applied	Number of results
PubMed	“Artificial intelligence”, “Machine learning”, “Deep learning”, “Artificial neural networks”, “Atrial Fibrillation”, “AF diagnosis”	10 Feb 2024	English language, full text, human subjects	68
Google Scholar	“Artificial intelligence”, “AI in AF detection”, “Machine learning in AF risk management”, “AI models for AF prediction”	10 Feb 2024	English language, full text, peer-reviewed	43

Study Selection

To be included, the study had to meet the following criteria: utilize AI technology, including machine learning (ML) and deep learning (DL); report measurable outcomes such as sensitivity, specificity, predictive accuracy, or diagnostic performance related to AF detection and management; have complete datasets; focus on human subjects; and have to be published in English. Studies combining AI with non-AI methods were included as long as the contribution of AI to the measurable outcomes was explicitly detailed. Exclusion criteria included studies not involving AI-based technology, lacking measurable outcomes, published in non-English languages, or focused on animal or in-vitro models. Duplicate records were identified and removed using EndNote reference management software.

The selection process was conducted independently by two reviewers, AP and SY. Disagreements during the selection process were resolved by a third reviewer, PS, through discussion and consensus. The titles of the articles obtained in the initial search were analyzed to determine if they covered the subject of study of this analysis. The abstracts of the remaining articles were then studied to establish the relevance of the given articles to the current study, such that they tried to answer the questions posed herein. At this point, the articles that passed the described eligibility criteria were then fully read to determine their utility and significance towards achieving the goal of systematic review (Table 2).

**Table 2:** Summary of study screening process.

Stage	Number of studies
Records identified from PubMed and Google Scholar	111
Records after duplicates and before screening	97
Records screened for incomplete data and abstract-only articles	97
Full-text articles sought for retrieval	90
Studies excluded based on relevance	27
Total studies Included in Review	39

Data Extraction and Outcome Measures, Quality Appraisal 

Quality appraisal was conducted independently by two reviewers, AP and SY, using the JBI critical appraisal checklist for qualitative research to ensure methodological rigor and reduce bias [20]. Discrepancies in scoring were resolved through discussion and, when necessary, adjudicated by a third reviewer, PS. During the process, duplicate studies were removed. An analysis was done on the titles and then the abstracts of each article obtained in the initial search to ensure that they reported on the primary outcomes delineated for this review. Hereafter, the articles that were left read entirely. The articles had to meet a minimum requirement by responding "yes" to at least 80% of the JBI assessment questions. The JBI critical appraisal checklist was chosen for its suitability in evaluating diverse methodologies, ensuring congruence between research questions, methodology, and data interpretation, which aligns with the scope of this review. The quality appraisal was done on thirty-nine papers, and all were included. The appraisal process is illustrated in Table 3.

**Table 3:** Results of quality appraisal on studies using the JBI checklist for qualitative studies. The term "Item" refers to the specific criteria from the JBI critical appraisal checklist for qualitative research. Each Item represents an essential aspect of study quality being assessed, such as study design, data analysis, or risk of bias. The checklist includes the following criteria: Item 1: Is there congruity between the research methodology and the research questions or objectives? Item 2: Is there congruity between the research methodology and the data collection methods? Item 3: Is there congruity between the research methodology and the representation and analysis of the data? Item 4: Is there congruity between the research methodology and the interpretation of results? Item 5: Is there a clear statement of findings? Item 6: Is the research method appropriate to address the research question? Item 7: Are ethical considerations clearly addressed? Item 8: Is there a clear statement on potential conflicts of interest? Item 9: Is there adequate representation of participants' voices in the findings? Item 10: Are the conclusions drawn from the findings appropriate? The total score for each study is based on how many of the 10 criteria were met, with a "1" indicating that the item was met, and a "0" indicating that it was not met.

Author(s) and year	Item 1	Item 2	Item 3	Item 4	Item 5	Item 6	Item 7	Item 8	Item 9	Item 10	Total
Andersen et al., 2017 [21]	1	1	1	1	1	1	1	0	1	1	9
Asgari et al., 2015 [22]	1	1	1	1	1	1	1	0	1	1	9
Baek et al., 2023 [23]	1	1	1	1	1	1	1	0	1	1	9
Bonini et al., 2022 [24]	1	1	1	1	1	1	1	0	1	1	9
Christopoulos et al., 2020 [25]	1	1	1	1	1	1	1	0	0	1	8
Gruwez et al., 2023 [26]	1	1	1	1	1	1	1	0	1	1	9
Guo et al., 2021 [27]	1	1	1	1	1	1	1	0	1	1	9
Hill, et al., 2020 [28]	0	1	1	1	1	1	1	0	1	1	8
Hill et al., 2019 [11]	1	1	1	1	1	1	1	0	1	1	9
Hill et al., 2022 [29]	1	1	1	1	1	1	1	0	1	0	9
Hill et al., 2020 [30]	1	1	1	1	1	1	1	0	1	1	9
Holmes et al., 2024 [31]	1	1	1	1	1	1	1	0	1	1	9
Isaksen et al., 2022 [32]	1	1	1	1	1	0	1	0	1	1	8
Kaminski et al., 2022 [33]	1	1	1	1	1	1	1	0	1	1	9
Lawin et al., 2022 [34]	1	1	1	1	1	1	1	0	1	1	9
Lee et al., 2022 [35]	1	1	1	1	1	0	1	0	1	1	8
Liu et al., 2022 [36]	1	1	1	1	1	1	1	0	1	1	9
Luo et al., 2021 [37]	1	1	1	1	1	1	1	0	1	1	9
Ma et al., 2023 [38]	1	1	1	1	0	1	1	0	1	1	8
Manetas-Stavrakakis et al., 2023 [39]	1	1	1	1	1	1	1	0	1	1	9
Müller et al., 2023 [40]	1	1	1	1	1	1	1	0	1	1	9
Ng et al., 2022 [41]	1	1	1	1	1	1	1	0	1	1	9
Poh et al., 2023 [42]	1	1	1	1	1	1	1	0	1	1	9
Prabhakararao E et al., 2022 [43]	1	1	0	1	1	1	1	0	1	1	8
Predel et al., 2020 [44]	1	1	1	1	1	1	1	0	1	1	9
Rabinstein et al., 2021 [45]	1	1	1	1	1	1	1	0	1	1	9
Rizwan et al., 2021 [46]	1	1	0	1	1	1	1	0	1	1	8
Rizwan et al., 2018 [47]	1	1	1	1	1	1	1	0	1	1	9
Santala et al., 2021 [48]	1	1	1	1	1	1	1	0	1	1	9
Schnabel et al., 2022 [49]	1	1	0	1	1	1	1	0	1	1	8
Sehrawat et al., 2022 [50]	1	1	1	1	1	1	1	0	1	1	9
Tiwari et al., 2020 [51]	1	1	1	1	1	1	1	0	1	1	9
Tran et al., 2023 [52]	1	1	1	1	1	1	1	0	1	1	9
Wasserlauf et al., 2019 [53]	1	1	1	1	1	1	1	0	1	1	9
Wegner et al., 2022 [54]	1	1	1	0	1	1	1	0	1	1	8
Wu et al., 2021 [55]	1	1	1	1	1	1	1	0	1	1	9
Xiong et al., 2022 [56]	1	1	1	1	1	1	1	0	1	1	9
Zhang et al., 2024 [57]	1	1	1	1	1	1	1	0	1	1	9
Zimmerman et al., 2023 [58]	1	1	1	1	1	1	1	0	1	1	9

Results

Search Results

The flowchart (Figure 1) illustrates our study selection process. We identified 111 studies, of which 39 were selected. All 39 studies were included in the review (Figure 1) (Table 4).

**Figure 1:** PRISMA flow diagram for the included studies

**Table 4:** Characteristics of the included studies. MT-DCNN: multi-task deep convolutional neural network, (CHADS2): congestive heart failure, hypertension, age ≥75 years, diabetes, and stroke; CHADS-VASc: congestive heart failure, hypertension, age ≥75years, diabetes, stroke, vascular disease; SVM: support vector machine.

Author(s) and year	Study design	Study objective	Outcomes
Andersen et al., 2017 [21]	Prospective study	A novel approach for AF detection based on inter-beat intervals	The proposed approach for AF detection based on Inter Beat Intervals (IBI) extracted from long-term electrocardiogram (ECG) recordings requires the detection of R-peaks in the ECG signal but allows for significantly reduced computation time without loss of performance.
Asgari et al., 2015 [22]	Prospective study	Novel method for automatic AF detection using wavelet transform and SVM	AF detection using Stationary Wavelet Transform and Support Vector Machine (SVM) has high accuracy, sensitivity, and specificity for AF detection.
Baek et al., 2023 [23]	Retrospective cohort study	To validate an AI-enhanced ECG algorithm for predicting PAF	An area under the receiver operating characteristic curve will be created to test and validate the datasets and assess the AI-enabled ECGs acquired during the sinus rhythm to determine whether AF is present.
Bonini et al., 2022 [24]	Review	Review of mHealth solutions in AF	mHealth devices are promising instruments in specific populations, such as post-stroke patients, to promote an early arrhythmia diagnosis in the post-ablation/cardioversion period, allowing checks on the efficacy of the treatment or intervention.
Christopoulos et al., 2020 [25]	Observational study	Develops an AI algorithm applied to electrocardiography during sinus rhythm to predict future AF	The AI-ECG may offer a means to assess risk with a single test and without requiring manual or automated clinical data abstraction.
Gruwez et al., 2023 [26]	Clinical study	Large-scale smartphone-based screening for AF	Smartphone-based AF screening is feasible on a large scale. Screening increased OAC uptake and impacted therapy of both new and previously diagnosed clinical AF but failed to impact risk factor management in subjects with subclinical AF.
Guo et al., 2021 [27]	Validation study	Develop an ML-based model for predicting AF onset in a population at high risk of incident AF.	The PPG-based ML model demonstrated a good ability to predict AF in advance. (Mobile Health [mHealth] technology for improved screening, patient involvement, and optimizing integrated care in atrial fibrillation; ChiCTR-OOC-17014138).
Hill et al., 2020 [28]	Clinical trial	To assess the effectiveness of this risk prediction algorithm combined with diagnostic testing for the identification of AF in a real-world primary care setting.	There is potential for the risk prediction algorithm to be implemented throughout primary care to narrow the population considered at highest risk for AF who could benefit from more intensive screening for AF.
Hill et al., 2019 [11]	Retrospective, cohort study	To develop and evaluate novel and conventional statistical and machine learning models for risk-predication of AF.	The optimal time-varying machine learning model exhibited greater predictive performance than existing AF risk models and reflected known and new patient risk factors for AF.
Hill et al., 2022 [29]	Clinical study	To assess the effectiveness of a machine learning risk-prediction algorithm in conjunction with diagnostic testing for identifying undiagnosed atrial fibrillation (AF) in primary care in England.	The AF risk-prediction algorithm accurately identified high-risk participants in both arms. While the proportions of AF and related arrhythmia diagnoses were not significantly different between high-risk arms, intervention arm participants who underwent diagnostic testing were twice as likely to receive arrhythmia diagnoses compared with routine care. The
Hill, et al., 2020 [30]	Validation study	To assess the cost-effectiveness of targeted screening, informed by a machine learning (ML) risk prediction algorithm, to identify patients with A	Targeted screening using an ML risk prediction algorithm has the potential to enhance the clinical and cost-effectiveness of AF screening, improving health outcomes through efficient use of limited healthcare resources.
Holmes et al., 2024 [31]	Review	To evaluate an artificial intelligence (AI)-enabled ECG algorithm to predict AF detected by PCT after index stroke.	Clinical scores, including CHA2DS2-VASc and CHARGE-AF, can risk stratify patients but lack desired accuracy.
Isaksen et al., 2022 [32]	Review	reviews the state of the art of machine learning algorithms for the detection, prediction, and management of atrial fibrillation (AF)	The prediction of paroxysmal or future AF currently operates at a level of precision that is too low for clinical use. Further studies are needed to determine whether patient selection for interventions may be possible with machine learning.
Kaminski et al., 2022 [33]	Retrospective cohort study	To evaluate the ability of an AI algorithm to predict incident AF in an emergency department cohort of patients presenting with palpitations without concurrent AF.	The AI-ECG algorithm predicted AF with an AUC of 0.74 (95% CI 0.68-0.80), an optimum threshold with sensitivity of 79.1% (95% Confidence Interval (CI) 66.9%-91.2%), and a specificity of 66.1% (95% CI 63.6%-68.6%).
Lawin et al., 2022 [34]	Review	To discuss the advances in digital health applications for the detection of AFib	The overall evidence for an improvement in hard clinical endpoints and positive effects on clinical care from the use of DiHA in the setting of AFib is scarce.
Lee et al., 2022 [35]	Validation study	To propose a deep learning system for early detection of atrial enlargement or fibrillation using Convolutional Recurrent Neural Networks and Parallel Bi-directional Long Short-Term Memory Networks.	The more ECG data collected in the exercise phase are involved, the more effective our system is in diagnosis of the diseases.
Liu et al., 2022 [36]	Validation study	To investigate the feasibility of using photoplethysmography signals and a deep convolutional neural network to classify multiclass arrhythmia types.	This study demonstrated the feasibility of classifying multiclass arrhythmias from photoplethysmography signals using deep learning techniques.
Luo et al., 2021 [37]	Validation study	To investigate the feasibility of using photoplethysmography signals and a deep convolutional neural network to classify multiclass arrhythmia types.	Classifying multiclass arrhythmias from photoplethysmography signals using deep learning techniques is attractive for population-based screening and may hold promise for the long-term surveillance and management of arrhythmia.
Ma et al., 2023 [38]	Review	To describe the status of AF monitoring technology using IoT and AI	Through ambulatory ECG measurement and intelligent detection technology, the probability of postoperative recurrence of AF can be reduced, and personalized treatment and management of patients with AF can be realized.
Manetas-Stavrakakis et al., 2023 [39]	Meta-analysis	To review the diagnostic accuracy of AI-based methods for the diagnosis of atrial fibrillation.	Our analysis showed that AI-based methods for the diagnosis of atrial fibrillation have high sensitivity and specificity for the detection of AF.
Müller et al., 2023 [40]	Prospective cohort study	To compare the efficacy and safety of two different high-power, short-duration ablation approaches for symptomatic AF.	High-power short-duration AF ablation with a target AI of 400 for non-posterior wall and 300 for posterior wall lesions resulted in comparable long-term results compared to higher AI (450/350) ablations with significantly lower risk for thermal.
Ng et al., 2022 [41]	Prospective multicenter study	To evaluate the performance of a wrist-worn device with lead-I ECG and continuous photoplethysmography for AF detection and burden estimation.	The field is still nascent, and several barriers will need to be overcome, including prospective validation in large, well-labeled data sets and more seamless information technology-based data collection/integration, before AI can be adopted into broader clinical EP practice.
Poh et al., 2023 [42]	Prospective cohort study	evaluated the performance of a wrist-worn device with lead-I ECG and continuous photoplethysmography (Verily Study Watch) and photoplethysmography	Continuous monitoring using a photoplethysmography-based convolutional neural network incorporated in a wrist-worn device has clinical-grade performance for AF detection and burden estimation.
Prabhakararao et al., 2022 [43]	Comparative study	MT-DCNN is compared with the state-of-the-art rhythm-based, rhythm- and morphology-based approaches.	A multi-task deep convolutional neural network (MT-DCNN) can accurately estimate the AF burden from long-term ECG recordings; thus, it has the potential to be used in remote patient monitoring applications for improved diagnosis, phenotyping, and management of AF.
Predel et al., 2020 [44]	Ethical analysis	to analyze the ethical challenges associated with screening for atrial fibrillation using smartwatches.	As smartwatches provide only a little information about the possible consequences, informed consent cannot be assumed. Ethical implementation could be archived if doctors provide smartwatches to patients who have been shown to benefit from them. The implementation and education should be managed by the doctor.
Rabinstein et al., 2021 [45]	Prospective cohort study	To determine if an AI-enabled ECG model can differentiate between patients with ESUS and those with known causes of stroke	AI-ECG may help guide the use of prolonged ambulatory cardiac rhythm monitoring in patients with ESUS to identify those who might benefit from anticoagulation.
Rizwan et al., 2021 [46]	Review	a discussion on all these aspects related to AF auto-diagnosis	There is a dire need for low-energy and low-cost but accurate auto-diagnosis solutions for the proactive management of AF.
Rizwan et al., 2018 [47]	Review	To provide an algorithm for accurate, automated detection of atrial fibrillation (AF) from ECG signals.	Feature selection and ensemble learning can be used to improve the performance of ECG-based classification of AF.
Santala et al., 2021 [48]	Validation study	evaluated the feasibility and accuracy of a wearable automated mHealth arrhythmia monitoring system	A consumer-grade, single-lead ECG heart belt provided good-quality ECG for rhythm diagnosis. The mHealth arrhythmia monitoring system, consisting of heart-belt ECG, a mobile phone application, and an automated AF detection, achieved AF detection with high accuracy, sensitivity, and specificity.
Schnabel et al., 2022 [49]	Observational study	Machine learning methods for predicting incident AF and AF post-stroke	ICD-coded clinical variables selected by machine learning can improve the identification of patients at risk of newly diagnosed AF. Using this readily available, automatically coded information can target AF screening efforts to identify high-risk populations in primary care and stroke survivors.
Sehrawat et al., 2022 [50]	Review	Role of AI-enabled ECG in AF detection and management	Algorithms using AI to interpret ECGs in various new ways have been developed. While still, much work needs to be done, these technologies have shown enormous potential in a short span of time. With further advancements and continuous research, these novel ways of interpretation may well become part of everyday clinical workflow.
Tiwari et al., 2020 [51]	Observational study	Machine learning approaches for identifying AF risk from EHR data	Machine learning approaches to electronic health record data offer a promising method for improving risk prediction for incident AF, but more work is needed to show improvement beyond standard risk factors.
Tran et al., 2023 [52]	Observational study	Impact of false AF alerts from wearables on older patients	A promising approach to avoid negative impact of false alerts is to employ artificial intelligence driven algorithms to improve accuracy.
Wasserlauf et al., 2019 [53]	Observational study	identifying cardiac arrhythmias and noise in ECG recordings	Without employing a time-consuming feature engineering step, the ensemble classifier trained with this architecture provided a robust solution to the problem of detecting cardiac arrhythmia from noisy ECG signals.
Wegner et al., 2022 [54]	Clinical study	Comparison of AF-sensing watch with insertable cardiac monitor for AF detection	An AF-sensing watch is highly sensitive for detection of AF and assessment of AF duration in an ambulatory population when compared with an ICM. Such devices may represent an inexpensive, noninvasive approach to long-term AF surveillance and management.
Wu et al., 2021 [55]	Review	Review of machine learning and neural networks in AF detection and management	Machine learning applications may aid cardiologists in the management of patients with already diagnosed atrial fibrillation by identifying patients at a high risk of recurrence after catheter ablation.
Xiong et al., 2022 [56]	Clinical study	predicting AF from ECG using ensemble learning	In feature extraction, this paper combined P-wave morphology parameters and heart rate variability parameters as input parameters for model training and validated the value of the combination of the proposed parameters for the improvement of the model’s predicting effect. In the calculation of the P-wave morphology parameters, the hybrid Taguchi-genetic algorithm was used to obtain more accurate Gaussian function fitting parameters. The prediction model was trained using the stacking ensemble learning method so that the model accuracy had better results, which could further improve the early prediction of atrial fibrillation.
Zhang et al., 2024 [57]	Clinical study	mAFA III pilot cohort study for structured follow-up rehabilitation packages in AF patients	Ancillary analyses determine the impact of the ABC pathway using smart technologies on the outcomes among the "high-risk” population (e.g., ≥75 years old, with multi-morbidities, with poly-pharmacy) and the application of artificial intelligence machine-learning AF risk prediction management in assessing AF recurrence.
Zimmerman et al., 2023 [58]	Report	To demonstrate the ability of AI approach to improve the accuracy and equity of stroke risk prediction.	Current risk stratification approaches are blind to social determinants of health, which are important modifiers of clinical variables and, ultimately, stroke risk. While effective stroke-prevention strategies are available, optimal implementation of these treatments is limited by (1) rudimentary stroke risk stratification tools (i.e., CHADS2-VA2Sc), and (2) disparities in care and outcomes of AF. There remains a critical need for personalized, socially aware, and equitable stroke risk prediction for patients with AF.

Study Characteristics

19 articles reported on AF risk stratification and twenty articles reported on AF risk management.

AI in AF Risk Stratification

Risk factors needed to train AI models for AF risk prediction include male sex, hypertension, previous heart failure, heart disease, and chronic kidney disease [45,48]. These predictors have demonstrated reliability for training machine learning models. However, additional predictors can be identified by machine learning from ICD codes to facilitate effective risk prediction in outpatient care [48]. Zimmerman et al. contend that existing risk stratification models such as CHADS2-VA2Sc are restricted and rudimentary, ignoring key risk factors such as social health determiners [58]. Machine learning models utilizing standard health record features generally perform better than traditional risk stratification models like CHADS2-VASc. For instance, the Observational Medical Outcomes Partnership Common Data Model achieved an area under the receiver operating characteristic curve (AUC) of 0.800, compared to a crude logistic regression model with an AUC of 0.794. This slight improvement in AUC indicates better discrimination between high- and low-risk patients, which can lead to more accurate and personalized clinical decision-making [51].

Despite reliability concerns of available risk predictors, certain AI risk stratification models, such as the optimal time-varying machine learning model, have demonstrated outstanding performance over conventional statistical models like Cox regression [11]. For instance, in the PULsE-AI trial involving 26,183 patients, ML models achieved AUCs of 0.653 for stroke prediction and 0.677 for major bleeding prediction, compared to 0.587 and 0.537 for CHADS2 and HAS-BLED scores, respectively [50,59]. These improved metrics translate to better discrimination between high- and low-risk patients, enhancing clinical decision-making by providing more accurate risk stratification. Notably, the former model validated the traditional risk factors and demonstrated the potential utility of novel factors such as pulse pressure and body mass index (BMI) changes [11]. The PULsE-AI trial validated the utility of a machine learning risk-prediction algorithm using diagnostic tests to determine the accuracy of identified high-risk participants [29]. A prediction model trained with the stacking ensemble learning method showed excellent prediction accuracy [55]. Similarly, AI-enabled electrocardiography (AI-ECG) surpassed cohorts for aging and research in genomic epidemiology-AF (CHARGE-AF) score in utility, requiring a single test to assess risk. However, Holmes et al. contend that current machine-learning algorithms lack the precision necessary for AF prediction and management [31]. Key challenges in applying ML models for AF care include data heterogeneity, which can lead to inconsistent performance across populations; lack of external validation, limiting their generalizability; opacity of ML algorithms, reducing clinician trust; and biases in training datasets, potentially exacerbating health disparities for underrepresented groups [31].

AI-Assisted Clinical Management

The application of AI in AF practice is dependent on large clinical studies in risk assessment and subsequent risk management. However, such studies require external validation of their high accuracy. As such, the efficacy of AI is tied to the models' attributes, input data quality, and the validation process. Nevertheless, there is still sufficient opportunity for further development and improvement of the current AI solutions. The research methods also need to be standardized so that AI solutions are validated by prospective studies, data sets are adequately tagged, and all data is handled responsibly [40].

AF risk of recurrence is linked to several factors, including age and left atrium (LA) size. Recurrence risk can be managed through targeted therapeutic interventions such as high power for short duration (HPSD) ablation for pulmonary vein isolation at index settings [40]. Comorbidity management, facilitated through AF detection using inter beat intervals (IBI) ECG data, is crucial for the management of AF burden [21]. Early detection of AF through IBI analysis allows for prompt initiation of anticoagulation therapy, reducing the risk of stroke in patients with AF. The REVEAL AF study demonstrated that insertable cardiac monitors (ICMs) detecting previously unknown AF led to changes in clinical management, including the initiation of oral anticoagulation in 63% of patients with detected AF [60]. Smartphone-based devices allow for self-heart rate monitoring. Such devices are more effective among the high-risk population, such as post-stroke patients [24]. Large-scale smartphone-based screening fails to improve risk factor management in subjects with subclinical AF [26]. Long-term and continuous AF monitoring can be afforded by wrist-worn wearables for the management of AF [41]. However, smartwatch screening presents ethical challenges unless the doctor-patient relationship is preserved and protected. Additionally, adherence to smartwatch-based monitoring can be challenging, especially for high-risk populations like post-stroke patients, who may face physical and cognitive impairments that limit consistent use [43,45,49]. AI can effectively discriminate false alerts, thus improving accuracy [50]. 

A deep learning system to distinguish between atrial enlargement and AF is productive for diagnosis [35]. Deep learning models, such as the convolutional recurrent neural network (CRNN) and parallel Bi-directional long short-term memory network (BiLSTM), can analyze P-wave parameters from exercise ECGs to differentiate between atrial enlargement and AF with high precision. This approach enhances the detection of atrial myocardial diseases, which are often precursors to AF, thereby enabling earlier and more accurate diagnosis. Ambulatory heart rate monitoring using AI-equipped devices can mitigate the risk of postoperative AF recurrence [37]. Similarly, a convolutional neural network (CNN) allowed the accurate detection of cardiac arrhythmia from noisy ECG signals [52]. CNNs enable accurate detection of cardiac arrhythmia from noisy ECG signals by automatically extracting relevant features, suppressing noise, utilizing multi-scale analysis, incorporating temporal information, and employing optimization techniques to handle class imbalances [61]. Machine learning facilitates the identification of patients at a high risk of recurrence after catheter ablation [55]. Its novel and disruptive capabilities can transform medical practices, potentially assisting cardiologists in managing patient care more effectively [57]. Similarly, an AI-enabled ECG algorithm can predict AF detected by prolonged cardiac telemetry after index stroke [30]. An ML-based model trained on a population at high risk of AF had high prediction accuracy [27]. Classifying multiclass arrhythmias from photoplethysmography signals using deep learning techniques is attractive for population-based screening and may hold promise for the long-term surveillance and management of arrhythmia [35]. AI-ECG may help guide the use of prolonged ambulatory cardiac rhythm monitoring in patients with embolic strokes of unknown source (ESUS) to identify those who might benefit from anticoagulation [44].

Discussion

This review sought to determine the utility of AI in AF prediction and management. The findings indicate that machine learning models are the main AI applications in AF risk stratification. AI-ECG models such as the optimal time-varying machine learning model and observational medical outcomes partnership common data model outperform existing models such as Framingham, ARIC, CHADS2-VA2Sc and CHARGE-AF score both in sensitivity and specificity parameters. Furthermore, wearable devices such as a patch monitor and a smartwatch are both a cost-effective and noninvasive alternative to insertable cardiac monitors for continuous monitoring and patient-oriented AF risk management. Wearable devices are particularly useful among high-risk populations, including postoperative and diagnosed patients.

Risk stratification is a crucial component of the integrated approach to AF management. It facilitates the assessment of potential future AF events, the probability of adverse outcomes, and the personalization of interventional strategies. Risk stratification involves identifying factors that predict the probability of AF occurrence. Machine learning models have been used to determine the most significant risk factors, which include male sex, hypertension, previous heart failure, heart disease, and chronic kidney disease [45,47]. However, as AI technology advances, additional predictors, such as social health determiners, are being identified [58]. This is possible as AI models continue to analyze larger and larger datasets, thus providing a more comprehensive risk assessment [11]. Such comprehensive assessments permit a more personalized approach to risk assessments compared to traditional models.

Risk management is also a key facet of integrated AF care. It is facilitated by AI-enabled wearable and mHealth solutions, which provide real-time AF detection and monitoring [41,53]. These devices allow for continuous ECG measurement to monitor the likelihood of postoperative AF recurrence [58]. Continuous monitoring using photoplethysmography AI-enabled devices has demonstrated accuracy that is clinically applicable [53,58]. Convolutional neural networks (CNN) enable the integration of electronic health records, imaging data, and historical data to improve the accuracy of risk assessments [52]. mHealth solutions can play a role in real-time risk assessment updates. Thus facilitating timely interventions and modification of treatment plans to prevent adverse events.

Deep neural networks have been used to predict AF ECG [23] and determine the association between risk management and AF clinical outcomes. As such, for patients undergoing catheter ablation, DNN can assist in the planning phase by analyzing photoplethysmography signals and identifying optimal ablation targets [35,36,54]. This personalized approach improves the probability of successful therapeutic interventions. AI models can predict the likelihood of procedural success or potential complications, aiding in shared decision-making and allowing for more informed discussions between healthcare providers and patients [33,34,39]. Furthermore, AI systems integrated with wearables and mHealth solutions can provide real-time analysis of patient data, including heart rhythm, allowing for prompt detection of treatment response or potential complications.

AI has tremendous potential in all fields; for example, it is being used to predict cardiogenic shock as well as screening for aortic stenosis [62,63]. Machine learning has immense disruptive potential for AF prediction and management; however, wearable and mHealth solutions present ethical challenges. Beneficence and non-maleficence need to be assured given the influence of private companies, privacy protection, liability, and doctor-patient-relationship. Prabhakararao et al. report that there is currently no evidence supporting better outcomes and reduced AF complications due to smartwatch use. Furthermore, smartwatches are plagued with false-positive results, which can cause harm [43]. Nevertheless, a novel convolutional denoising autoencoder (CDA) was able to effectively discriminate false alerts in wrist-based wearables [50]. As such ML tools retain the promise of accurate risk stratification and management. Despite these promises, wrist-based wearables are cost-prohibitive to many patients, thus raising the concern of equitable AF care [58]. Nevertheless, targeted screening using an ML risk prediction algorithm has the potential to enhance the cost-effectiveness of AF risk management, improving health outcomes through the efficient use of limited healthcare resources [29]. However, ML solutions must demonstrate significant performance improvements over standard risk-scoring models to encourage their adoption [50]. Furthermore, there is a concern about data quality, and biased AI models trained on unrepresentative datasets may result in biased predictions [40]. Models trained on data from specific demographics may not apply well to other populations, leading to disparities in performance across different ethnicities, age groups, or geographic regions [40]. As such, the efficacy of AI is tied to the model's attributes, input data quality, and the validation process. Nevertheless, there is still sufficient opportunity for further development and improvement of the current AI solutions. The research methods also need to be standardized so that AI solutions are validated by prospective studies, data sets are adequately tagged, and all data is handled responsibly [40]. 

Notably, most of the included studies are retrospective analyses, thus the reported AI models may perpetuate existing biases present in healthcare data, potentially resulting in inconsistency in the results [40,49,58]. There is an evident lack of reliable prospective validation studies, thus hindering the assessment of the real-world effectiveness and generalizability of these models [40,48]. The use of patient data in AI applications raises concerns about privacy and security. Ensuring compliance with data protection regulations and maintaining patient confidentiality should be the foundational tenets of AI solutions in AF care [23,43]. Data collected from patient records include baseline demographics, comorbidities, laboratory findings, echocardiographic findings, hospitalizations, and related procedural outcomes, such as AF ablation and mortality. However, efforts are being made to address these concerns. Such efforts include de-identification of ECG data through data encryption and anonymization [23]. Addressing these challenges requires collaboration between clinicians, statisticians, policymakers, and regulatory bodies. Strategies such as transparent model development, diverse and representative training datasets, and ongoing monitoring of AI performance can contribute to overcoming these limitations and facilitating the responsible integration of AI into AF care.

Limitations

This review has several limitations. The included studies varied in design, encompassing retrospective cohorts, validation studies, and clinical trials. These variations may introduce biases, such as selection bias in retrospective studies, and affect the generalizability and consistency of the findings. Additionally, the models were adapted differently by authors, including variations in feature selection methods, training datasets, or input variables, which may influence performance comparability and reproducibility. The lack of standardized methodologies further complicates direct comparisons across studies. Data quality remains a concern, with biases in training datasets and limited representativeness of populations, potentially reducing the applicability of the findings to diverse clinical settings. Future validation efforts could benefit from statistical approaches such as meta-analyses, sensitivity analyses, and subgroup evaluations to enhance the robustness of the conclusions.

## Conclusions

The findings indicate that ML-enabled devices and AI-ECG models have excellent sensitivity and specificity for AF prediction and management applications. Furthermore, AI-based devices can be convenient and non-invasive tools for AF management thus allowing long-term passive monitoring. However, further validation studies need to be conducted. Future research efforts should focus on the standardization of research methods, systematic data set labeling, and maintaining patient confidentiality. Furthermore, further studies are necessary to evaluate the cost-effectiveness, risks, and benefits of AI solutions in integrated AF care.
